The article "Predictive Value Analysis of Serum Ig A, Ig G, and TNF-α in Recurrence of Multiple Myeloma" was published in 2022. Journal: Dis Markers.

# Predictive Value Analysis of Serum Ig A, Ig G, and TNF-*α* in Recurrence of Multiple Myeloma

**DOI:** 10.1155/2022/2095696

**Published:** 2022-10-12

**Authors:** Xinyan Jia, Xiangxin Liu, Wenzhong Yang

**Affiliations:** ^1^Department of Hematology, Shanghai East Hospital, Tongji University School of Medicine, Shanghai 200120, China; ^2^Department of Hematology, Ji'an Hospital of Shanghai East Hospital, Ji'an, 343000 Jiangxi, China; ^3^Department of Hematology, Shanghai Punan Hospital of Pudong New District, Shanghai 200125, China

## Abstract

**Objective:**

The study is aimed at analyzing the predictive value of serum Ig A, Ig G, and TNF-*α* in the recurrence of multiple myeloma (MM).

**Methods:**

136 patients with MM treated in our hospital from January 2010 to January 2017 were followed up for 5 years. Finally, 100 patients who met the inclusion and exclusion criteria and had the complete follow-up visit were selected as the study subjects, with the recurrence of MM as endpoint event, and the observation was taken until the occurrence of endpoint event in patients or the termination of this study. They were divided into the recurrence group (RG) and the nonrecurrence group (NRG) according to whether the endpoint event occurred. The venous blood of patients was collected at the first diagnosis and subsequent visit (at the time of recurrence or termination of the study) to measure the Ig A and Ig G using a full automatic special protein analyzer and the TNF-*α* level by enzyme-linked immunosorbent assay. The data obtained in this study were analyzed by univariate analysis to choose the factors with difference in statistical significance to draw the ROC curve, and the areas under the curve (AUC) were recorded to analyze the potential mechanism of Ig A, Ig G, and TNF-*α* in predicting the recurrence of MM.

**Results:**

After follow-up visit, there were 62 patients with recurrence (62.0%) and 38 patients without recurrence (38.0%), with no obvious difference in gender, age, body weight, and immune classification between the two groups (*P* > 0.05). Compared with the NRG, the levels of soluble interleukin-2 receptor (sIL-2R) and *β*_2_-microglobulin (*β*_2_-MG) in the RG at the first diagnosis were distinctly higher (*P* < 0.001); the levels of Ig A, Ig G, and TNF-*α* in the RG at the first diagnosis were visibly higher (*P* < 0.05); and the levels of Ig A, Ig G, and TNF-*α* in the RG at the subsequent visit were clearly higher (*P* < 0.05). There was a correlation between Ig G, Ig A, and TNF-*α* and *β*_2_-MG at the first diagnosis and the subsequent visit (*P* < 0.05); there was a correlation between Ig G and TNF-*α*, and sIL-2R at the first diagnosis and the subsequent visit (*P* < 0.05); and there was a correlation between Ig A and sIL-2R at the subsequent visit (*P* < 0.05). The AUC of Ig G, Ig A, and TNF-*α* in predicting the MM at the first diagnosis were 0.772, 0.776, and 0.778, respectively.

**Conclusion:**

The serum Ig A, Ig G, and TNF-*α* had a predictive value in the recurrence of MM, and TNF-*α* was correlated with sIL-2R and *β*_2_-MG, with the highest AUC and the best predictive value.

## 1. Introduction

Multiple myeloma (MM), as a malignant proliferative disease of bone marrow plasma cells, belongs to the category of B cell lymphoma, characterized by abnormal proliferation of plasma cells with the overproduction of monoclonal immunoglobulin or light chain (M protein) [1, 2], with no effective healing method at present. Patients still have a high possibility of recurrence after complete remission [3, 4], so that the system of recurrence prediction is very important in the prevention and treatment of MM. According to the immunoglobulin types secreted by myeloma cells, MM is divided into Ig A type, Ig G type, Ig M type, and light chain type in clinic, and further divided into *κ* type and *λ* type according to light chain type [5, 6]. There are differences in the secretion levels of immune factors and inflammatory factors in patients with different immune classifications, but patients can still find the same markers to evaluate the prognosis; for example, Dong Yi et al. have found that the expression of p53 protein, bcl-2 protein, and soluble interleukin-2 receptor (sIL-2R) in patients with MM at the first diagnosis and subsequent visit is positively correlated with *β*_2_-microglobulin (*β*_2_-MG), speculating that p53 protein, bcl-2 protein, and sIL-2R can be used to predict the recurrence of MM [7]. At present, there are a few reports to predict the recurrence of MM by immunoglobulin in academic circles, but it is known that B cells have an interaction with T cells and natural cells, affecting the results of immune response through different mechanisms [8, 9], so that the immune factors and inflammatory factors can reflect the activation, development, and differentiation of B cells. In clinical practice, the factors related to B cells can be selected to evaluate the recurrence possibility of patients, and the relationship between Ig A, Ig G, and TNF-*α* and B cells has been confirmed by literature. Ig A and Ig G are synthesized by plasma cells differentiated from B cells, and TNF-*α* can promote B cell differentiation, which plays an important role in osteolytic destruction in patients with MM. Based on this, 100 patients with MM in complete remission after treatment were followed up in this study to analyze the relationship between the levels of Ig A, Ig G, and TNF-*α* and the recurrence of MM to establish a good predictive mechanism in clinic.

## 2. Materials and Methods

### 2.1. Study Design and Case Selection

As a retrospective study, 100 patients who met the requirements of experimental design were selected as the study subjects finally to analyze the predictive value of serum Ig A, Ig G, and TNF-*α* in the recurrence of MM (see the technical route in Figure 1). The inclusion criteria are the following: (1) Patients were in line with the diagnostic criteria of Chinese guideline for diagnosis and treatment of multiple myeloma (2013) [10]. (2) Patients were treated for the first time and had a complete remission after treatment. (3) Patients were treated in the hospital in the whole process, with complete clinic information. (4) The age of patients exceeded 18 years old. The exclusion criteria are the following: (1) patients with the hearing impairment, language disorders, unconsciousness, and mental illness, and patients who cannot communicate with others; (2) patients who withdrew the treatment halfway; (3) patients with no complete remission after treatment [11]; (4) patients with the bacterial and viral infection at the first diagnosis; (5) patients with the dysfunction of vital organs such as heart, brain, liver and kidney; (6) patients with other organic diseases; (7) patients with incomplete clinic information; and (8) patients with no complete follow-up visit in the whole process.

### 2.2. Moral Consideration

This study met the principles of Declaration of Helsinki (2013) [12], and patients and their families who were aware of the purpose, significance, content, and confidentiality of the study signed informed consent.

### 2.3. Methods and Observation Indices

100 patients with MM in complete remission after treatment who were treated in our hospital from January 2010 to January 2017 were selected to collect the data of social demography and clinical manifestation at the first diagnosis. The data of social demography included gender, age, and body weight of patients, and the data of clinical manifestation included immune classification, clinical stage, and the levels of serum sIL-2R, *β*_2_-MG, Ig A, Ig G, and TNF-*α*. The fasting venous blood of patients (3 ml) was taken in the morning at the first diagnosis to obtain the serum after centrifugation to determine the levels of serum sIL-2R and TNF-*α* by enzyme-linked immunosorbent assay (Beijing Kewei Clinical Diagnostic Reagent Inc.; NMPA approval No.: S20060028), the *β*_2_-MG level by radioimmunoassay method (Tianjin Xiehe Pharmaceutical Science and Technology Co., Ltd., NMPA approval No.: S20083085), and the levels of Ig A and Ig G by a full automatic special protein analyzer (Bio-Rad Laboratories, Inc.; original matching reagent; NMPA (I) 20182220158).

All patients were followed up for 5 years, mainly outpatient follow-up, supplemented by telephone follow-up, with the recurrence of MM as the endpoint event (recurrence referred to the recurrence after complete remission of primary treatment), and the observation was taken until the occurrence of endpoint event in patients or the termination of study. They were divided into the recurrence group (RG) and the non-recurrence group (NRG) according to whether the endpoint event occurred. The fasting venous blood of patients was taken again at the subsequent visit (at the time of recurrence or termination of the study) in the morning to determine the levels of Ig A, Ig G, and TNF-*α*, and then, the univariate analysis was performed on the levels of Ig A, Ig G, and TNF-*α* at the first diagnosis and subsequent visit. For the factors with difference in statistical significance, the occurrence of endpoint event was assigned to 1, and no occurrence of endpoint event was assigned to 0. The ROC curve was drawn by SPSS20.0 to record the areas under the curve (AUC) to analyze the value of Ig A, Ig G, and TNF-*α* in predicting the recurrence of MM.

### 2.4. Statistical Treatment

In this study, the data processing software was SPSS20.0, and the GraphPad Prism 7 (GraphPad Software, San Diego, USA) was used to draw the pictures. The items included in the study were enumeration data and measurement data tested by *X*^2^ test and *t* test. *P* < 0.05 indicated that the difference was statistically significant.

## 3. Results

### 3.1. Comparison of Baseline Data in Patients

Except for the level values of sIL-2R and *β*_2_-MG at the first diagnosis, there was no significant difference in other baseline data between the two groups (*P* > 0.05), as shown in Table 1.

### 3.2. Comparison of Levels of Ig A, Ig G, and TNF-*α* in Patients at the First Diagnosis and Subsequent Visit

Compared with the NRG, the levels of Ig G, Ig A, and TNF-*α* in the RG at the first diagnosis were visibly higher (48.18 ± 34.95 vs 33.71 ± 25.46, 22.98 ± 28.01 vs 10.60 ± 16.01, 6.50 ± 1.13 vs 5.30 ± 0.93, *P* < 0.05), and the levels of Ig G, Ig A, and TNF-*α* at the subsequent visit in the RG were clearly higher (51.60 ± 35.57 vs 33.31 ± 25.74, 27.65 ± 32.84 vs 9.81 ± 14.91, 7.97 ± 0.95 vs 4.14 ± 0.42, *P* < 0.05). See the levels of Ig A, Ig G, and TNF-*α* in patients with different immune classifications at the first diagnosis and subsequent visit in Table 2.

### 3.3. Correlation Analysis between Ig A, Ig G, and TNF-*α*, and sIL-2R and *β*_2_-MG in Patients at the First Diagnosis and Subsequent Visit

There was a correlation between Ig G, Ig A, and TNF-*α*, and *β*_2_-MG at the first diagnosis and the subsequent visit (*P* < 0.05); there was a correlation between Ig G and TNF-*α*, and sIL-2R at the first diagnosis and the subsequent visit (*P* < 0.05); and there was a correlation between Ig A and sIL-2R at the subsequent visit (*P* < 0.05), as shown in Table 3.

### 3.4. Value of Ig A, Ig G, and TNF-*α* in Predicting the Recurrence of MM

The AUC of Ig G, Ig A, and TNF-*α* in predicting the MM at the first diagnosis were 0.772, 0.776, and 0.778, respectively. See variable assignment in Table 4 and the ROC curve in Figure 2.

## 4. Discussion

B cells are derived from pluripotent stem cells of bone marrow, which can be differentiated into plasma cells under antigen stimulation, and plasma cells can synthesize and secrete the antibody (immunoglobulin), affecting the immunoglobulin levels in patients [13], so that multiple myeloma patients with malignant proliferation of plasma cells have an obviously abnormal immunoglobulin level, suggesting that the immunoglobulin level can reflect the differentiation and activation of plasma cells [14, 15]. The study of domestic scholars Feige et al. on 66 patients with Ig G-type MM has shown that patients with Ig G ≤64 g/L are distinctly superior to patients with Ig G >64 g/L in terms of overall survival and progression-free survival [16], which further confirmed that the abnormal immunoglobulin level was an intuitive reflection of monoclonal hyperplasia degree in MM, as an indicator to evaluate the disease state and reflect the degree of tumor load. At present, there is a lack of literature in analyzing the prognosis of patients with MM from the related factors of B cells, but the potential value of immunoglobulin in predicting the recurrence of MM cannot be ignored. In this study, after five years of follow-up visit, there were 62 patients with recurrence (62.0%) and 38 patients without recurrence (38.0%), and the levels of sIL-2R, *β*_2_-MG, Ig A, Ig G, and TNF-*α* in the RG at the first diagnosis were signally higher than those in the NRG (*P* < 0.001). *β*_2_-MG, as a classical marker for evaluating the clinical stage of patients with MM in the ISS, exists on the serous membrane of all karyocytes, and it involves in the surface identification of lymphocytes and the killing of cell receptors [17, 18]. Because *β*_2_-MG can reflect the proliferation rate of myeloma cells, some studies use it as a state variable to test the value of related indicators in evaluating prognosis, and indicators that are significantly related to *β*_2_-MG can be used to test the severity of patients with MM [19, 20]. R analysis results showed that there was a correlation between Ig G, Ig A, and TNF-*α*, and *β*_2_-MG at the first diagnosis (*P* < 0.05); that is, high levels of Ig G, Ig A, and TNF-*α* were independently correlated with high *β*_2_-MG level. The higher the *β*_2_-MG level at the first diagnosis, the higher the levels of Ig G, Ig A, and TNF-*α*, and the higher the possibility of recurrence after complete remission, with a consistency of the overall trend and the results of related factors analysis. Ig G, as a classical indicator to reflect the B cell status, is commonly used in the studies related to immune [21, 22]. Liu et al. have believed that low Ig G level is associated with B cell dysfunction, while high Ig G level reflects that the rate of B cell differentiation into plasma cells is accelerated and the total number of plasma cells is increased [23]. Ig A accounts for 10%–20% of the total serum immunoglobulins, which has a predictive value in children with nephrotic syndrome, clostridium difficile-associated diarrhea, and other recurrent diseases. However, this study found that there was a correlation between Ig G and TNF-*α* and sIL-2R at the first diagnosis and the subsequent visit (*P* < 0.05), with no correlation between Ig A and sIL-2R at the first diagnosis. sIL-2R, as an immunosuppressive factor that reflects the tumor burden, can compete with the membrane to bind interleukin-2 (IL-2), hindering the important biological response regulated by IL-2, making the cellular immune dysfunction of body, and eventually leading to the cells with malignant clone escaping from immune surveillance to have an excessive proliferation. In this study, sIL-2R is also a state variable, which has been confirmed to be associated with the recurrence of MM. Therefore, the determination of Ig G, Ig A, and TNF-*α* at a specific time can be used to infer the level changes of *β*_2_-MG and sIL-2R, thus evaluating the prognosis of patients.

ROC analysis further showed that the AUC of Ig G, Ig A, and TNF-*α* in predicting the MM at the first diagnosis were 0.772, 0.776, and 0.778, respectively, suggesting that the predictive value of TNF-*α* is higher than that of Ig G and Ig A, and the relationship between TNF-*α* and B cells has been confirmed in the literature. This marker can promote the proliferation of B cells and lymphocytes and accelerate the rate of B cells differentiation into plasma cells [24]. Moreover, the structure outside the cell membrane of TNF receptor type I (TNF-R1) and receptor type II is homologous, and the former can enter the blood circulation after the abscission of cell membrane. Yuhua et al. have found that the TNF-*α* level in patients with MM is signally higher than that in normal control group, and with the increase of clinical stages, the TNF-*α* level shows a progressive tendency in ladder type, suggesting that TNF-*α* is related to tumor load in patients with MM, and this marker reflects the biological parameters of tumor load [25]. Yuhua has further proposed that the growth of MM is regulated by TNF-*α*, and MM can be treated in clinic by inhibiting TNF-*α* to act on related signaling pathways. The above results showed that TNF-*α* was an important serum marker in the diagnosis, treatment, and prognosis of MM and had a high clinical reference value.

It is worth noting that this study only included patients with MM who had complete remission after initial treatment. Affected by practical factors, only 100 patients received the complete follow-up visit, with small study samples. Subsequent studies need to further increase the sample size to support the above conclusions, and enrich the system of immune factors and inflammatory factors related to B cells to predict the MM.

## 5. Conclusion

In recent years, the application of new targeted drugs like proteasome inhibitor and immunomodulator has prolonged the complete remission rate of patients with MM, but patients are still unable to cure, and most patients still relapse after systematic treatment, even ushering in a death ending. Since the recurrence mechanism of MM is not clear, it is important to establish an effective prediction mechanism of recurrence. In this study, 100 patients with MM were followed up, founding that there was an obvious difference in the levels of serum Ig A, Ig G, and TNF-*α* between recurrent and non-recurrent patients, and the three indicators were correlated with the classical index (*β*_2_-MG) of MM, with the AUC ≥ 0.7. Therefore, the serum Ig A, Ig G, and TNF-*α* have a predictive value in the recurrence of MM, and TNF-*α* has the highest AUC and the best predictive value. In practice, the three indicators could be combined to evaluate the prognosis of patients comprehensively.

## Figures and Tables

**Figure 1:** Technical route.

**Figure 2:** ROC curve analysis of Ig A, Ig G, and TNF-*α* in predicting the recurrence of MM. Notes. The sources of curve in Figure 2 were Ig G (first diagnosis and subsequent visit), Ig A (first diagnosis and subsequent visit), TNF-*α* (first diagnosis and subsequent visit), and reference line, while the vertical axis represented the sensitivity, and the lateral axis represented 1-specificity.

**Table 1:** Comparison of baseline data between the two groups.

Items	RG (*n* = 62)	NRG (*n* = 38)	*x* ^2^/*t*	*P*
Gender			0.020	0.887
Male	35 (56.45)	22 (57.89)		
Female	27 (4355)	16 (42.11)		
Age ($\bar{\text{x}}\pm \text{s}$, years)	55.37 ± 5.19	55.76 ± 5.29	0.427	0.670
Body mass ($\bar{\text{x}}\pm \text{s}$, kg)	66.21 ± 5.32	66.75 ± 5.24	1.061	0.282
Immune classifications				
Ig A type	14 (22.58)	11 (28.95)	0.509	0.475
Ig G type	38 (61.29)	22 (57.89)	0.113	0.737
Ig M type	2 (3.23)	1 (2.63)	0.029	0.866
Light chain type	8 (12.90)	4 (10.53)	0.126	0.723
Clinical stage				
Stage I	1 (1.61)	3 (7.89)	2.421	0.120
Stage II	18 (29.03)	13 (34.21)	0.295	0.587
Stage III	43 (69.35)	22 (57.89)	1.360	0.244
sIL-2R at the first diagnosis ($\bar{\text{x}}\pm \text{s}$, ng/L)	0.80 ± 0.07	0.56 ± 0.08	6.119	<0.001
*β*_2_-MG at the subsequent visit ($\bar{\text{x}}\pm \text{s}$, mg/L)	6.22 ± 1.07	4.94 ± 0.99	15.084	<0.001
Complications				
Hypertension	13 (20.97)	7 (18.42)	0.096	0.757
Diabetes mellitus	6 (9.68)	3 (7.89)	0.124	0.725
Treatment methods				
Chemotherapy	21 (33.87)	14 (36.84)	0.091	0.762
Immunomodulator	14 (22.58)	9 (23.68)	0.016	0.899
Radiotherapy	25 (40.32)	12 (31.58)	0.773	0.379
Others	2 (3.23)	3 (7.89)	1.081	0.298

**Table 2:** Comparison of levels of Ig A, Ig G, and TNF-*α* in patients with different immune classifications at the first diagnosis and subsequent visit.

Groups	*n*	Ig G (g/L)		Ig A (g/L)		TNF-*α* (ng/L)	
		First diagnosis	Subsequent visit	First diagnosis	Subsequent visit	First diagnosis	Subsequent visit
Ig A type							
RG	14	5.05 ± 1.23	6.52 ± 0.24	74.28 ± 8.53	88.32 ± 2.21	6.41 ± 1.02	8.01 ± 1.23
NRG	11	3.97 ± 0.42	3.21 ± 0.43	35.21 ± 5.68	32.68 ± 5.68	5.21 ± 0.98	4.08 ± 0.24
*t*		2.777	24.444	13.057	39.156	2.970	10.397
*P*		0.011	<0.001	<0.001	<0.001	0.007	<0.001
Ig G type							
RG	38	75.18 ± 10.42	79.68 ± 5.10	8.32 ± 0.21	10.32 ± 2.21	6.54 ± 1.20	7.98 ± 0.80
NRG	22	55.11 ± 5.65	54.98 ± 5.32	0.60 ± 0.05	0.52 ± 0.08	5.34 ± 0.98	4.12 ± 0.50
*t*		8.333	17.796	169.107	20.716	3.980	20.401
*P*		<0.001	<0.001	<0.001	<0.001	<0.001	<0.001
Ig M type							
RG	2	4.30 ± 0.04	5.95 ± 1.20	6.65 ± 0.01	8.38 ± 0.05	6.43 ± 1.21	7.58 ± 0.84
NRG	1	3.24	2.54	0.20	0.18	5.40	4.31
*t*		21.637	2.320	526.640	133.905	0.695	3.179
*P*		0.029	0.259	0.001	0.005	0.613	0.194
Light chain type							
RG	8	6.40 ± 0.45	8.51 ± 0.65	6.91 ± 0.78	8.62 ± 0.67	6.48 ± 0.98	7.99 ± 1.01
NRG	4	5.42 ± 0.20	4.57 ± 0.65	0.50 ± 0.06	0.48 ± 0.04	5.31 ± 0.48	4.36 ± 0.24
*t*		4.081	9.898	16.019	23.695	2.219	6.932
*P*		0.002	<0.001	<0.001	<0.001	0.051	<0.001

**Table 3:** Correlation analysis between Ig A, Ig G, and TNF-*α*, and sIL-2R and *β*_2_-MG in patients at first diagnosis and subsequent visit.

Groups	Time	sIL-2R (g/L)		*β*_2_-MG (g/L)	
		*r*	*P*	*r*	*P*
Ig G (g/L)	First diagnosis	0.225	0.024	0.213	0.033
	Subsequent visit	0.242	0.016	0.209	0.037
Ig A (g/L)	First diagnosis	0.167	0.096	0.247	0.013
	Subsequent visit	0.216	0.031	0.298	0.003
TNF-*α* (g/L)	First diagnosis	0.440	<0.001	0.235	0.019
	Subsequent visit	0.823	<0.001	0.501	<0.001

**Table 4:** Variable assignment.

Variables	Variable assignment	AUC
Endpoint events	Occurrence = 1 and no occurrence = 0	—
Ig G at first diagnosis	Variable assignment	0.788
Ig G at subsequent visit	Variable assignment	0.758
Ig A at first diagnosis	Variable assignment	0.748
Ig A at subsequent visit	Variable assignment	0.727
TNF-*α* at first diagnosis	Variable assignment	0.791
TNF-*α* at subsequent visit	Variable assignment	0.817

## Data Availability

Data to support the findings of this study is available on reasonable request from the corresponding author.
